# The Essential Role of FoxO1 in the Regulation of Macrophage Function

**DOI:** 10.1155/2022/1068962

**Published:** 2022-08-11

**Authors:** Shan Jie Rong, Chun Liang Yang, Fa Xi Wang, Fei Sun, Jia Hui Luo, Tian Tian Yue, Ping Yang, Qilin Yu, Shu Zhang, Cong-Yi Wang

**Affiliations:** ^1^The Center for Biomedical Research, Department of Respiratory and Critical Care Medicine, Key Laboratory of Pulmonary Diseases of Health Ministry, Tongji Hospital, Tongji Medical College, Huazhong University of Sciences and Technology, Wuhan, China; ^2^Department of Clinical Nutrition, Tongji Hospital, Tongji Medical College, Huazhong University of Sciences and Technology, Wuhan, China

## Abstract

Macrophages are widely distributed in various tissues and organs. They not only participate in the regulation of innate and adaptive immune response, but also play an important role in tissue homeostasis. Dysregulation of macrophage function is closely related to the initiation, development and prognosis of multiple diseases, including infection and tumorigenesis. Forkhead box transcription factor O1 (FoxO1) is an important member among the forkhead box transcription factor family. Through directly binding to the promoter regions of downstream target genes, FoxO1 is implicated in cell proliferation, apoptosis, metabolic activities and other biological processes. In this review, we summarized the regulatory role of FoxO1 in macrophage phagocytosis, migration, differentiation and inflammatory activation. We also emphasized that macrophage reciprocally modulated FoxO1 activity via a post-translational modification (PTM) dominant manner.

## 1. Introduction

The forkhead box O (FoxO) protein family consists of four major members in mammals, namely FoxO1, FoxO3a, FoxO4 and FoxO6. They are distinct in tissue distribution and regulatory function while sharing a common DNA binding domain, which can recognize the cis-element of “TTGTTTAC” motif [1]. FoxO1, the first transcription factor identified in the FoxO family, is widely expressed in different tissues and organs. Activated FoxO1 translocates into the nucleus, where it regulates the transcription of various downstream molecules, including molecules relevant to cell cycle arrest, autophagy associated genes, metabolic enzymes and immune mediators. However, once FoxO1 becomes sequestered in the cytoplasm, it can no longer exert its regulatory function.

There is compelling evidence that FoxO1 is implicated in the regulation of adaptive immune response. It has been noted to be essential for the homeostasis of naïve T cell repertoire by up-regulating the surface expression of interleukin-7 receptor-alpha [2, 3]. Therefore, genetic ablation of FoxO1 in T cells exacerbates the severity of inflammatory bowel disease (IBD) along with enhanced T cell activation and effector T cell (Teff) differentiation in mice [4]. Specifically, FoxO1 hinders Teff polarization but favors the program of regulatory T cell (Treg) cells [5]. FoxO1 promotes the generation, suppressive capability as well as the phenotypic stability of Treg cells, by enhancing the expression of master transcription factor Foxp3 and other functional genes such as *CTLA-4* [6–8]. Meanwhile, FoxO1 can directly bind to the DNA binding domain of *RORγt* to inhibit its transcriptional activity, thereby impairing the generation of Th17 cells [9]. On the other hand, inactivation of FoxO1 promotes terminal differentiation of memory CD8^+^ T cell by up-regulating the expression of T-bet [10] . Takeshi et al. demonstrated that after germinal center formation, silencing of FoxO1 resulted in the disruptive migration of B cells from the light zone to the dark zone, and this process was mediated by the down-regulation of transcription factor BATF [11]. Compared to the well-recognized function in adaptive immune system [12], the role of FoxO1 in innate immune cells, especially in macrophages, is less appreciated.

Macrophages, as a major innate cell type present essentially in all human tissues, are derived from either embryonic progenitors (tissue resident macrophages) or bone marrow precursors and peripheral blood monocytes (bone marrow derived macrophages) [13]. Other than their role in immune responses, macrophages also exert a prominent effect on tissue homeostasis by regulating non-hematopoietic cell types [14]. Particularly, FoxO1-dependent regulation of macrophage functionality has been recognized to be complicated in multitudinous disease conditions such as infection, metabolic disorders, fibrosis, autoimmune diseases and tumor development [1, 15–21]. Therefore, in this review, we sought to update the advancement of FoxO1 as an important molecular switch in macrophage function and discuss how macrophages dynamically adjust their function by altering FoxO1 activity primarily through post-translational modifications.

## 2. FoxO1 Enhances Macrophage Phagocytic and Migratory Activity

Macrophage phagocytosis plays a critical role in tissue homeostasis under both physiological and pathological conditions. Apoptotic bodies and the resulting cell debris generated from normal tissue turn-over are timely engulfed by resident macrophages, thereby avoiding secondary necrosis to induce inflammatory responses [22, 23]. Macrophages actively probe and clear invading pathogens to defend the body against infectious diseases. Insufficient macrophage phagocytosis predisposes to the initiation and development of various diseases. Critically, FoxO1 strengthens the phagocytic capacity of macrophages via different approaches [24] (Figure 1). On the one hand, FoxO1 directly fosters the expression of *GATA6* [13], which renders macrophages to possess phagocytic function [25]; on the other hand, FoxO1 promotes autophagosome formation to accelerate the processing of phagocytosed materials [26], and autophagy has been proposed as a mechanism by which macrophages deal with intracellular pathogens [27]. In line with these observations, Foxo1 deletion led to a marked reduction in autophagy [22].

The migratory capacity of macrophages is an essential supplement for the optimal implementation of the phagocytic activity. Once tissue homeostasis is perturbed, patrolling macrophages are recruited to the damaging area to assist in the phagocytic process. Subsequently, after ingesting the antigens, some macrophages are able to migrate to the draining lymph nodes, where they serve as potent antigen-presenting cells. C-C motif chemokine receptor 2 *(CCR2)*, a member of G protein-coupled receptor, is recognized as a vital mediator of macrophage migration. FoxO1 has been demonstrated to directly bind to a small nucleotide region between −291 and−208 in the mouse *Ccr2* promoter, by which it enhances *Ccr2* transcription, leading to reinforced macrophage migration [28].

## 3. FoxO1 Fosters Macrophage Differentiation Program

Depending on the varied microenvironment, macrophages exhibit tremendous plasticity and exist in distinct activation state. According to the specific transcriptional factor and cytokine profiling, macrophages are classified into M1 subset (canonically activated macrophage) induced by LPS and/or IFN-*γ* and M2 subset (alternatively activated macrophage) elicited by IL-4 or IL-10 [29, 30]. Although such dichotomization seems oversimplified, it provides valuable insight into the mechanistic understanding of macrophage differentiation and function (Figure 1). More recently, the role of FoxO1 in macrophage polarization has aroused increasing attention. Studies demonstrated that activated FoxO1 skews macrophage towards M1 phenotype through directly binding to the promoter regions of MHCII and IL-1*β* [31, 32]. Activation of SIRT1 pathway upon LPS/IFN-*γ* stimulation enhances FoxO1 expression to drive pro-inflammatory cytokine secretion [33]. Moreover, engagement of TLR4 further activates FoxO1 which in turn boosts M1 lineage via the IRF3 pathway [17]. Intriguingly, other than the positive regulatory effect on M1 polarization, FoxO1 is also found to be essential in M2 commitment. MSC derived TGF-*β* can enhance the nuclear translocation of FoxO1 via suppressing Akt signaling pathway and predispose macrophage to M2 fate, thereby reducing macrophage inflammatory response and elevating the phagocytic ability [34, 35]. Indeed, there is evidence that FoxO1 up-regulates the expression of IL-10, which is critical for both M2 induction and effector function [15]. IRF4, a key transcription factor in macrophage metabolism, can also be augmented by FoxO1 [36]. However, it remains unclear why FoxO1 exerts opposite roles in macrophage differentiation and whether co-factors exist to dictate the direction of FoxO1 functional outcome.

## 4. FoxO1 Promotes Macrophage Inflammasome Activation

Reactive oxygen species (ROS), consisting of superoxide anion, hydrogen peroxide, hydroxyl free radical and nitric oxide, are a group of chemical substances with active property and strong oxidative activity. In macrophage, ROS are majorly produced in mitochondria where NADPH oxidase and peroxidase are the two responsible catalytic enzymes. In order to maintain the steady state of ROS system, excessive ROS can be eliminated by the buffering anti-oxidative components such as Superoxide dismutase (SOD) catalase, glutathione peroxidase and ascorbic acid. Once the balance breaks down, accumulation of ROS occurs, which facilitates inflammasome formation, leading to the secretion of pro-inflammatory cytokines such as IL-18 and IL-1*β* [19]. Cyclophilin D, a regulator of mitochondrial permeability transition, accelerates LPS-induced mitochondrial ROS production in a FoxO1 dependent manner [37]. Similarly, upon activation FoxO1 drives the transcription of IL-1*β* [19]. Collectively, those data support that FoxO1 likely serves as an important link bridging ROS accumulation and inflammasome activation.

## 5. FoxO1 Is Tightly Regulated in Macrophages

Given the indispensable roles in macrophage function, FoxO1 needs to be finely controlled for proper activity. Compared to the regulation at transcriptional level, post-translational modification (PTM) is regarded as the main form of FoxO1 regulation in macrophages [26].

### 5.1. Phosphorylation

FoxO1 has three conserved phosphorylation sites, including Thr24, Ser256 and Ser319 [38]. The phosphorylation level of FoxO1 is negatively correlated with the functional activity. Activated/dephosphorylated FoxO1 translocates into the nucleus and modulates the transcription of downstream genes. Nevertheless, phosphorylation inhibits the function of FoxO1 by promoting the nuclear exportation and subsequent protein degradation [38]. PI3K/AKT signaling pathway is identified as the major upstream regulator. It has been reported that miR-142-5p, which directly targets on PTEN, promotes the osteoclastogenesis of bone marrow-derived macrophages through elevating the phosphorylation level of FoxO1 [39]. Besides, Dong et al. revealed that lithium upregulated phosphorylated FoxO1 expression by activating PI3K/Akt signaling in microglial cells, resulting in inhibition of toll-like receptor 4 expression [40].

### 5.2. Acetylation

Protein acetylation is dynamically controlled by histone/protein acetyltransferases (HATs) and histone/protein deacetylases (HDACs). The Sirtuin family, a class of NAD-dependent deacetylase belonging to HDACs, contains seven members (SIRT1-7) that have quite different subcellular localization as SIRT1, SIRT2, SIRT6, SIRT7 are mainly distributed in the nucleus, SIRT1 and SIRT2 can also appear in the cytoplasm while SIRT 3-5 primarily locate in the mitochondria [20, 33]. Deacetylation of FoxO1 is essential for its nuclear translocation and functional activity, and SIRTs are its key epigenetic regulators in macrophage. SIRT1 is involved in FoxO1 deacetylation as ablation of SIRT1 unleashes FoxO1 and impairs the G1/S transition to blunt macrophage self-renewal [41]. Another study pointed out that SIRT1 deacetylated FoxO1 to repress osteoclast formation by activating the ATP6vOd2/Cathepsin signaling pathway. SIRT3 mediated deacetylation of FoxO1 was indicated to potentiate M2 polarization, which plays a role in inhibiting the formation of renal calcium oxalate crystals [42]. In addition, increased acetylated FoxO1 was reported to enhance macrophage activation and migration toward synoviocyte-derived chemo-attractants when myeloid Sirt6 was deficient [20].

### 5.3. Ubiquitination

The ubiquitination process involves a series of reaction mediated by ubiquitin activating enzyme E1, ubiquitin conjugating enzyme E2 and ubiquitin ligase E3. Frequently, ubiquitination of FoxO1 works in coordination with protein phosphorylation and acetylation. For example, phosphorylation leads to an increased nuclear exportation of FoxO1. After that, FoxO1 is ubiquitinated and subsequently degraded by cytoplasmic proteasomes. On the other hand, the acetylation level of FoxO1 is negatively correlated with ubiquitination. Loss of SIRT6 in macrophage elicits enhanced FoxO1 acetylation along with reduced FoxO1 ubiquitination [20]. Despite numerous reports identified the degrading role of FoxO1 ubiquitination, direct evidence regarding to the engaged E1/E2/E3 enzymes and the sites for ubiquitin attachment remains scarce and further research is undoubtedly required.

## 6. Discussion

Studies on FoxO1 provide evidence for its important roles in the regulation of macrophage function. FoxO1 gives an impetus to macrophage phagocytosis, migration and activation in different ways. However, the role of FoxO1 in macrophage polarization is still controversial. For instance, in acute lung injury model, up-regulation of FoxO1 triggered by HMGB1 treatment promotes the expression of inflammatory cytokines like TNF-*α* and IL-1*β* [43]. FoxO1 was reported to support M1 program and power the expression of pro-inflammatory factors by binding to the promoter regions of CCR2, IL-1*β* or MHCII [28, 31, 32]. Meanwhile, another studies show that FoxO1 is also able to fuel the M2 phenotype by elevating the level of IL-10 and IRF4 [36]. The regulation of macrophage polarization is complicated and the polarization is the result of multiple factors. Most studies merely focused on *in vitro* polarized M1 or M2 macrophage, and also, the classification of M1 and M2 is too simple to represent all the characteristics of macrophages. So, it is an issue of concern to reconcile such apparent conflicting observations and whether additional co-factors of FoxO1 exist to help dictate the functional outcome of FoxO1 remains to be defined.

Undoubtedly, the proper regulation of FoxO1 activity, especially through post-translational modification (PTM), is essential for macrophage function. PTMs including phosphorylation, acetylation and ubiquitination affect FoxO1 nuclear translocation and the transcriptional activity (Figure 2). However, the involvement of other forms of PTM and the related catalytic enzymes should not be ignored. Arginine methylation, catalyzed by protein arginine methyl transferases (PRMTs), is an important protein modification that participates in various cellular processes such as gene expression regulation, DNA repair and protein-protein interaction. Cellular experiments have demonstrated that PRMT1 methylates FoxO1 primarily at Arg248 and Arg250, and methylated FoxO1 abrogates Akt-induced phosphorylation of FoxO1 at Ser253, which in turn contributes to enhanced nuclear localization and decreased protein degradation [44, 45]. However, relevant study of FoxO1 methylation in macrophage is limited and so does the case of other PTM forms.

The protein expression and modifications of FoxO1 could be greatly altered under a variety of disease conditions including infection, ischemic reperfusion injury (IRI), allergic asthma, obesity and tumorigenesis (Table 1). Dysregulation of macrophage phagocytosis, migration, polarization and inflammasome activation affects the progression and prognosis of such diseases. A great number of researches have shown that targeted deletion of FoxO1 using FoxO1-selective inhibitor AS1842856 or genetic ablation approach in macrophages attenuates the development of asthmatic lung inflammation by down-regulating IRF4 mediated M2 macrophage polarization [36, 46]. However, loss function of FoxO1 in macrophage exacerbates tumor growth via suppressing the expression of MHCII [32]. In conclusion, FoxO1 is tightly and differentially controlled under distinct disease settings. At present, the functional studies on FoxO1 are mainly performed on animals and cells, and relevant clinical studies are bare. In future clinical research and drug development, immunotherapy based on the regulation of macrophage function by FoxO1 may be a good research direction.

## Figures and Tables

**Figure 1:** Schematic diagram for the regulatory effect of FoxO1 on macrophage. (a) The role of FoxO1 in macrophage polarization. SIRT1 can promote the deacetylation of FoxO1 in the presence of LPS stimulation, which in turn accelerates nuclear translocation of FoxO1. FoxO1 skews macrophage towards M1 phenotype through binding to the promoter regions of MHCII and IL-1*β* directly. The other hand, FoxO1 up-regulates the expression of IL-10 and ADAR1, which is critical for M2 induction. FoxO1-driven IRF4 transcription promotes nuclear translocation of FoxO1 mediated by inhibiting PI3K-Akt signaling. (b) The function of FoxO1 in macrophage migration. Under oxidative stress, FoxO1 signaling is enhanced through JNK-MST1 pathway and facilitates CCR2 expression, leading to reinforced macrophage migration. (c) The effect of FoxO1 activity on macrophage phagocytosis. The expression of pro-phagocytotic factor GATA6 is upregulated by nuclear FoxO1, while the phosphorylation of FoxO1 hampers the nuclear translocation of FoxO1 following mTOR activation. (d) The impact of FoxO1 on macrophage inflammasome activation. Upon activation, FoxO1 drives the transcription of IL-1*β* and accelerates LPS-induced mitochondrial ROS production. FoxO1 also serves as an important link bridging ROS accumulation and inflammasome activation. *SIRT1, sirtuin1; ADAR1, adenosine deaminase acting on double-stranded RNA 1; MST1, Mammalian STE20-like kinase-1; CYPD, Cyclophilin D.*

**Figure 2:** Activity of FoxO1 is under tightly control in macrophage. Protein phosphorylation, acetylation and ubiquitination are the major post-translational modification forms that affect the expression level, subcellular distribution and the transcriptional activity of FoxO1. Phosphorylation, PI3K/AKT signaling pathway mediates the phosphorylation of FoxO1, whereas phosphorylation inhibits its function by promoting the nuclear exportation and subsequent protein degradation; Acetylation, Deacetylation of FoxO1 is essential for its nuclear translocation and functional activity during which process SIRTs are the key regulators in macrophage; Ubiquitination, the degradation of FoxO1 ubiquitination mainly dependents on ubiquitination in macrophages. The phosphorylation combined with acetylation and ubiquitination orchestrates FoxO1 function. The phosphorylation leads to an increased nuclear exportation of FoxO1, the exported FoxO1 is ubiquitinated and subsequently degraded in cytoplasmic proteasomes. On the contrary, the acetylation of FoxO1 fosters the nuclear transcription and negatively regulates the ubiquitination. *PML, Promyelocytic Leukemia Nuclear Bodies; SIRT6, sirtuin-6 (NAD-dependent protein deacetylase sirtuin-6).*

**Table 1:** Implications of FoxO1 in macrophage functional regulation under disease settings.

Manipulation	Upstream of FoxO1	FoxO1 activity	Effect on macrophage	Disease phenotype	Reference
*Chemical compounds*					
AS1842856	—	Inhibited	M2↓	Asthma↓	[36]
Ang- [1–7]	TLR4–JNK	Inhibited	M1↓	Inflammation ↓	[47]
AA	JNK	Inhibited	Proliferation↓	—	[48]
ATRA	RAR*α*	Inhibited	M2↑	Liver ischemia -reperfusion injury↓	[49]
ICG-001	*β*-Catenin	Enhanced	MMT↓	Kidney fibrosis↓	[21]
*Genetic (indirect)*					
*Nrf2 cKO*	Nrf2–Akt	Inhibited	M1↑	Liver ischemia -reperfusion injury↑	[50]
*CypD cKO*	—	Inhibited	M1↓	Inflammation ↓	[37]
*LysM-Irs2*	Akt		M2↓	Obesity↑	[18]
*LysM-Sirt6*	—	Enhanced	M1↑	Rheumatoid arthritis↑	[20]
*LysM-PTEN*	—	Inhibited	M1↓	Acute lung injury ↓	[43]
*PTEN* siRNA	Akt/*β*-catenin	Inhibited	M1↓	Liver ischemia -reperfusion injury↓	[51]
*CaMKKβ* siRNA	—	Enhanced	Autophagy↑	Anti-bacteria↑	[22]
*LKB1* vector	—	Enhanced	M1↑	Tuberculosis infection↓	[16]
*ADAR1* adenovirus	miR-21	Enhanced	M2↑	Allogeneic graft rejection↓	[34]
*Genetic (direct)*					
*LysM-FoxO1*	—	Inhibited	M2↑; M1↓	S. aureus infection↑	[23]
*LysM-FoxO1*	HIF-1*α*	Inhibited	M2↑	Tumor↑	[32]
*FoxO1* cKO	TLR4-PI3K-Akt	Inhibited	M1↓	Obesity↓	[17]
*FoxO1* shRNA	Insulin–Akt	Inhibited	Apoptosis↓	Obesity↓	[1]

Abbreviations: AS1842856, a pharmacologic inhibition of FoxO1; Ang, angiotensin; AA, arachidonic acid; ATRA, all-trans retinoic acid; RAR*α*, retinoic acid receptor *α*; ICG-001,a known inhibitor of *β*-catenin/TCF transcription by selectively blocking the *β*-catenin/CREB-binding protein interaction; MMT, macrophage–myofibroblast transition; Nrf2, nuclear factor erythroid 2-related factor 2; CypD, cyclophilin D; PTEN, phosphatase and tensin homologue; LKB1, liver kinase B1; ADAR1, adenosine deaminase acting on double-stranded RNA 1.

## Data Availability

All data generated or used during the study appear in the submitted article.
